This article has been retracted.

# Observation of the Effect of Nursing BPR on Thrombolytic Efficacy and Prognosis of Patients with Cerebral Infarction Based on CT Images

**DOI:** 10.1155/2022/3106904

**Published:** 2022-09-14

**Authors:** Shaomin Wang, Xiao Miao, Guanghui Zhang, Dandan Li, Li Xu

**Affiliations:** ^1^Neurology, The First Affiliated Hospital of Kangda College of Nanjing Medical University, Lianyungang 222002, Jiangsu, China; ^2^Neurosurgery, The First Affiliated Hospital of Kangda College of Nanjing Medical University, Lianyungang 222002, Jiangsu, China; ^3^Internal Medicine-Neurology, The First Affiliated Hospital of Kangda College of Nanjing Medical University, Lianyungang 222002, Jiangsu, China; ^4^The Department of Nursing, Kangda College of Nanjing Medical University, Lianyungang 222002, Jiangsu, China; ^5^Nursing Department, The First Affiliated Hospital of Kangda College of Nanjing Medical University, Lianyungang 222002, Jiangsu, China

## Abstract

Cerebral infarction has become the main cause of death among Chinese residents, especially ischemic cerebral infarction. The existing CT technology is not very effective for the detection of cerebral infarction, and some angiography has problems such as blurring and shadowing. In order to understand the treatment methods and effects of patients with cerebral infarction, this article observes the effect of nursing BPR on thrombolytic efficacy and prognosis of patients with cerebral infarction based on CT images. The patients were divided into thrombolytic group and nonthrombolytic group, and a simple rating scale was used to assess the motor function of the patients' limbs, and the stroke scale was used to assess the patient's neurological function. Compare the baseline data, the time of admission, 24 hours and 7 days, the scores before and after treatment, and the ratio between the two groups. According to the monitoring, record each time point. The analysis of the occurrence of primary endpoint was events and secondary endpoint events and risk factors affecting limb motor function. The results of the study found that, based on the computer scanning observation of nursing BPR, compared with the traditional model, the patient's bleeding was significantly reduced, and the time required for nursing was also reduced by more than 50% compared with the traditional model. Compared with the traditional nursing model, the satisfaction of patients with the BPR nursing model is nearly 40% higher than that of the traditional nursing model. This shows that the observation of thrombolytic effect in patients with cerebral infarction based on computed tomography and BPR nursing can produce good therapeutic effects.

## 1. Introduction

With the major changes in production and lifestyle brought about by the development of science and technology, ischemic stroke has become a major threat to people's health due to its high incidence, high disability, and high fatality rate. Intravenous thrombolytic therapy and intravascular interventional therapy have definite curative effects. In particular, intravenous thrombolytic therapy within a time window is safe and simple and is a first-line treatment method. However, intravenous thrombolysis also has some problems, such as increased incidence of hemorrhagic transformation after treatment, and individual differences in curative effects among patients. Previous studies have shown that it may be more logical to choose thrombolytic therapy based on imaging findings. Observing the impact can analyze the middle cerebral artery blood flow classification, occlusion location, pial collateral blood supply, right-to-left shunt, severe carotid artery stenosis or occlusion, the establishment of collateral circulation, ulcerative atherosclerotic plaque, and other factors that are related to the effect of intravenous thrombolysis in patients with middle cerebral artery occlusion and ischemic stroke. Because the etiological basis of cerebral thrombosis is mainly atherosclerosis, the factors that produce atherosclerosis are the most common causes of cerebral infarction. To explore these imaging characteristics, the effect of thrombolytic therapy and prognostic impact have been explored.

The continuous development of imaging provides the possibility for further research and exploration. At present, many studies are being carried out on the observation of the efficacy of thrombolytic therapy for cerebral infarction, and there are also many studies on the prediction and evaluation of the efficacy of intravenous thrombolysis by imaging methods. CT image observation can accurately show the course of large blood vessels and the blood flow filling in the lumen. It is currently the gold standard for the diagnosis of aneurysms, arteriovenous malformations, arterial stenosis or occlusion, and other vascular diseases. CT imaging observation and nursing BPR can find the lesion within 2 hours of the occurrence of cerebral infarction, which is much earlier than the conventional fast spin echo sequence. It plays an important role in early diagnosis and provides an important basis for early treatment.

For CT imaging observations, experts at home and abroad have done many studies. Zang et al. explore the dynamic changes of serum C-reactive protein (CRP), fibrinogen (FIB), and D-dimer (DD) to better characterize progress cerebral infarction. Carotid vascular ultrasound and neurological deficit scores were recorded. On admission, the carotid artery stenosis rate of the progressive group was significantly higher than that of the nonprogressive group [1]. Lee et al. passed a 59-year-old woman who spontaneously visited the emergency room due to subjective weakness on the right side. She was treated with dual antiplatelet drugs and aspirin. The MRI diffusion-weighted image showed acute infarction in the anterior cerebral artery area. This case showed acute infarction of CSAH. Rarely, it is necessary to work hard to determine the cause and consider antiplatelet drug therapy [2]. Aksu et al. take a blood sample from the patient before imaging to determine the level of copeptin. After imaging examination, the patients were divided into diagnostic groups, to determine the level of copeptin in patients with suspected intracranial events, and to determine whether the level of copeptin can be used for the identification of cerebral infarction, intracranial hemorrhage, and subarachnoid hemorrhage in the emergency room [3]. For cerebral infarction, there are also related studies. Ekingen et al. study included patients over 18 years of age who were diagnosed with cerebral infarction from December 2011 to November 2012. A total of 90 participants were included. The diagnosis of ischemic stroke through CCT and clinical findings was infarct patients and 50 healthy controls. The results showed that the levels of Galectin-3 and GFAP were significantly increased in ischemic stroke patients with normal CCT. In ROC curve analysis, 70.59% sensitivity and 70% specificity were detected [4]. Deveci et al. recruited patients with stable coronary artery disease (CAD) who received CAG with or without PCI. Compare the clinical and angiographic characteristics of patients with and without SECI. The risk of SECI after CAG and PCI increases with the complexity of CAD (represented by SS). SS is a predictor of SECI risk, and SECI is a complication that should be considered more often after CAG [5]. Cheng et al. explored the relationship between basal ganglia cerebral infarction and paroxysmal atrial fibrillation (PAF) caused by abnormal vagus nerve tone. Cases were divided into basal ganglia infarction group and nonbasal ganglia infarction group according to the anatomical location of cerebral infarction. The incidence of PAF in the basal ganglia infarction group was significantly higher than that in the nonbasal ganglia infarction group. The incidence of basal ganglia cerebral infarction was related to age. The incidence of PAF in the 79-year-old basal ganglia cerebral infarction group was significantly higher than that in the nonbasal ganglia cerebral infarction group [6]. Volny et al. believe that thrombolysis of cerebral infarction has been regarded as a successful angiography result. In order to illustrate the near-perfect angiographic results, the near-complete reperfusion category has been introduced. The patient received intravenous thrombolytic therapy. When stroke neurologists and neuroradiologists agreed to assess the results, the agreement increased to almost perfect [7]. These studies have provided some references for this article, but due to the lack of relevant experimental samples and the different experimental methods used, the experimental results are not reproducible.

In this article, the patients with cerebral infarction are grouped by CT image observation and nursing BPR, and the patients in different groups are observed, as well as observing the head and neck vascular sclerosis and ulcerative plaques, the establishment of collateral circulation, right to left shunt, etc. The method is scientific, feasible, and in line with ethical requirements. Based on the imaging observation, exploring the correlation between these factors and the effect of intravenous thrombolysis has certain theoretical value and practical significance.

## 2. Thrombolytic Efficacy and Prognostic Methods

### 2.1. Cerebral Infarction

Cerebral infarction, also known as ischemic stroke, refers to the stenosis or obstruction of the cerebral vascular lumen caused by atherosclerotic plaques or heart attacks in the cerebral arterial system, causing local arterial hemorrhage or cerebral artery stenosis, leading to ischemia. Hypoxic necrosis and irreversible damage of brain tissue occurred [8, 9]. The clinical manifestations are sudden consciousness disorder, physical disorder, speech disorder, and mental disorder. The peculiar physical symptoms of the disease lead to the peculiar psychological characteristics of the patient, which are mainly manifested as depression, loss of interest, deterioration of pessimism, irritability, lack of initiative, and general weakness. If these symptoms persist for more than 2 weeks, it is called poststroke depression (PSD). PSD is one of the common complications of stroke. It not only affects the recovery of nerve function and hinders the improvement of cognitive function, but also complicates the treatment of physical diseases. At the same time, it also prolongs the patient's hospital stay and increases medical expenses. The prognosis and rehabilitation of the disease can even make the patient think of suicide, which ultimately affects the patient's quality of life and increases the risk of death. Therefore, the treatment of cerebral infarction should pay special attention to patients with depression after the brain [10]. Cerebral infarction is divided into cerebral thrombosis, cerebral embolism, and lacunar cerebral infarction according to the different pathogenesis.

Because the sudden cerebrovascular accident brings more or less discomfort to the patient's daily life, the patient gradually develops emotional disorders, and neurological deficits lead to physical dysfunction. Clinical researchers at home and abroad are very concerned about stroke disease itself. At the same time, more and more attention has been paid to the psychological changes of patients after stroke. Most researchers believe that the relationship between myocardial infarction and depression is mutual. Cerebral infarction can cause depression, and persistent depression can also delay the recovery of brain nerve function in heart attack patients.

With the advancement of science, the research on the correlation of PSD is constantly deepening, but PSD is the result of the combined effect of exogenous and endogenous factors, and its influencing factors are complicated. The nursing staff is the patient's family member, and the low mRS score at the end of 3 months of onset and intravenous thrombolytic therapy are protective factors for PSD at the end of 3 months in patients with cerebral infarction, which can significantly reduce the incidence of PSD [11]. Different nursing staff (family nursing/nursing care) are related to the occurrence of depression after severe stroke at the end of 3 months in patients with cerebral infarction (especially in patients with cerebral infarction not treated by intravenous thrombolysis); the improvement of neurological function in patients with cerebral infarction at the end of 3 months is related to the 3. The occurrence of mild, moderate, and severe depression at the end of the month is related; the acute thrombolytic therapy in patients with cerebral infarction is associated with the occurrence of severe poststroke depression in patients with cerebral infarction at the end of 3 months. Therefore, it is recommended that medical staff consider patients with the above risk factors as high-risk groups for PSD, pay attention to mood swings, pay attention to psychological changes during stroke treatment, and diagnose and actively intervene in poststroke depression, such as strengthening emotional counseling, active communication, and when necessary supplemented with antidepressants that can effectively reduce psychological stress and relieve symptoms of patients [12]. 90% of the risk of cerebral infarction can be attributed to 10 simple risk factors, which are high blood pressure, smoking, excessive waist-to-hip ratio, poor diet, lack of physical exercise, diabetes, excessive alcohol consumption, excessive mental stress, and depression, having underlying heart disease and hyperlipidemia.

In recent years, as the average life expectancy of our country's population has increased, the number of patients with cerebral infarction has increased year by year. At present, for patients with cerebral infarction, antiplatelet aggregation agents or anticoagulants, free radical scavengers, brain protection agents, circulation improving drugs, and other drugs are widely used in clinical practice. Recombinant tissue fiber is used for patients with acute cerebral infarction who meet the indications for thrombolysis. Intervention with plasminogen activator is the most effective therapeutic drug. With the continuous advancement of medical methods and rehabilitation technology, the mortality rate of cerebral infarction is also slowly decreasing at a trend of 0.5% per year, but the disability rate has increased. Patients with neurological deficits lead to physical dysfunction and, at the same time, gradually develop mood disorders of varying degrees. Cerebral thrombosis is the most common type of cerebral infarction, accounting for about 60% of all cerebral infarctions, so the so-called “cerebral infarction” actually refers to cerebral thrombosis.

Motor dysfunction caused by acute cerebral infarction is one of the common clinical manifestations. The treatment of patients from supine position to standing will limit unnecessary muscle activity of the patient, activate the motor muscles with more active muscles, and apply the training content to life. Although it promotes the plasticity and reorganization of the brain, it is because factors such as weak muscle strength in patients with acute cerebral infarction make it difficult for patients to exercise actively [13, 14]. You can use manual contact, instructions, verbal communication, visual stimulation, etc. to inform the patient of the muscles that need to be exercised and provide assistance, so as to achieve the training of different muscles in the same exercise, improve the smaller muscle strength in the exercise mode, and gradually make the patient achieve independent completion of the corresponding tasks and achieve functional activities, and then through resistance exercises, the patients can stretch their muscles after exercise, reduce muscle fatigue, enhance muscle endurance, and restore motor function [15].

### 2.2. CT Imaging

Computed Tomography (CT), that is, electronic computed tomography, which uses precisely collimated X-ray beams, gamma rays, ultrasonic waves, etc., together with a highly sensitive detector, makes a cross-sectional scan around a certain part of the human body one by one. The basic principle of CT imaging is that when the continuous spectrum rays emitted by the ray tube penetrate the detected object, the attenuation coefficient of the penetrating material (that is, the radius and the absorption coefficient of the material at the radius are different) is detected. The difference in the internal penetration thickness will cause the light intensity of the transmitted object to be different [16]. This difference is recorded by the detector and displayed on the X-ray image in the form of gray-scale difference, which is the basic principle of CT scanning.

As shown in Figure 1, the structure of a typical CT imaging detection system is shown in the figure above. The system is composed of a radiation source, a high-voltage power supply, a radiation imaging device, a computer, and a display [17, 18]. The high-voltage power supply provides high-voltage to the ray source to drive the ray tube to generate rays. The ray imaging device converts invisible ray images into digital images, and the computer is responsible for image collection, processing, and display. According to the difference in the absorption and transmittance of X-rays by different tissues of the human body, a highly sensitive instrument is used to measure the human body, and then the data obtained by the measurement is input into the electronic computer. A cross-sectional or three-dimensional image of the inspected part of the human body is used to find small lesions in any part of the body.

Suppose that the thickness of the measured object is *T*, the average attenuation coefficient of X-rays in the material is *μ*, the size of the defect in the measured object in the X-ray transmission direction is Δ*T*, and the attenuation coefficient of the ray in the defect is *μ*′, and then, the relationship is as follows. The total intensity *I* of the ray is as follows:

(1) $$\begin{array}{c} I=I_{0}^{e-\mu }T\left(n+1\right). \end{array}$$

The above formula *I*_0_ is the initial intensity of incident X-rays, and *n* is the scattering ratio between X-rays and the object. The transmitted ray intensity of the nondefective part*I*_*p*_ is as follows:

(2) $$\begin{array}{c} I_{p}=I_{0}e^{-\mu T}. \end{array}$$

The transmitted ray intensity of the defect part*I*_*t*_ is

(3) $$\begin{array}{c} I_{t}=I_{0}e^{-\mu \left(T-\Delta T\right)-\mu^{\prime }\Delta T}. \end{array}$$

The ratio of the intensity difference between the transmitted X-rays of the defective part and the nondefective part to the background ray intensity *I* was

(4) $$\begin{array}{c} \frac{\Delta I}{I}=\frac{\left(e^{\left(\mu -\mu^{\prime }\right)\Delta T}-1\right)}{\left(n+1\right)}\approx \frac{\left(\mu -\mu^{\prime }\right)\mathrm{*\Delta}T}{\left(n+1\right)}. \end{array}$$

The radiation dose of CT diagnosis is larger than that of ordinary X-ray machines, so it is not suitable for pregnant women to perform CT examination. In the case that the radiation attenuation coefficient of the defective material *μ*′ is much smaller than the average attenuation coefficient *μ* of the inspected object, that is, the absorption of the radiation by the defective material is rarely negligible, then

(5) $$\begin{array}{c} \frac{\Delta I}{I}\approx \frac{\mu \Delta T}{\left(n+1\right)}. \end{array}$$

CT images are slice images, and cross-sections are commonly used. To visualize the entire organ, multiple consecutive slice images are required. Through the use of image reconstruction procedures on CT equipment, coronal and sagittal slice images can also be reconstructed, and the relationship between organs and lesions can be viewed from multiple angles. From the previous analysis, we can know that the difference in the spatial distribution of the ray intensity after the ray emitted from the ray tube passes through the object to be inspected is the fundamental source of image contrast in the radiographic inspection system. When using radiation to irradiate an object, the radiation passing through the object will be affected by the effect of the material and produce certain attenuation [19]. The attenuation changes with the density of the object, as shown in Figure 2.

When the object as a whole is an inhomogeneous substance, the attenuation coefficient at this time *μ* is no longer a specific value, but a function *μ*=*μ*(*x*, *y*). In a specific direction and path *L*, the attenuation of the rays can be expressed as

(6) $$\begin{array}{c} {\int^{}}_{L}\mu dl=In\left(\frac{I_{0}}{I}\right). \end{array}$$

Defining the attenuation value of a certain section as a generalized function*f*(*x*, *y*), the value of the line integral along the straight line *L* can be obtained:

(7) $$\begin{array}{c} p_{f}\left(s,\varphi \right)={\int^{}}_{L}f\left(x,y\right)dl. \end{array}$$

Rotate the coordinate system *xoy*. The rotation method is as follows: take the origin as the center *ϕ* and rotate the angle in the counterclockwise direction to obtain a new coordinate system *x*′*oy*′. At this time, the parameter equation of the straight line *L* is expressed *x*′*oy*′ as

(8) $$\begin{array}{c} \left\{\begin{array}{c} x=s\cos\phi -t\sin\phi \\ y=s\sin\phi +t\cos\phi \end{array}.\right. \end{array}$$

The function transformation relationship *x*′*oy*′ in the coordinate system *f*(*x*, *y*) can be obtained:

(9) $$\begin{array}{c} f\left(x,y\right)={\int^{}}_{-\infty }^{\infty }f\left(s\cos\phi -t\sin\phi ,s\sin\phi +t\cos\phi \right)dt. \end{array}$$

The internal information of the object to be measured is estimated through the collected projection data information, so as to realize the reconstruction of the object. The inversion formula of the transformation is

(10) $$\begin{array}{c} \hat{f}\left(r,\theta \right)=\frac{1}{2\pi^{2}}\frac{\partial p_{f}\left(s,\varphi \right)}{\partial s}dsd\varphi . \end{array}$$

Transform the expression to get the convolution form:

(11) $$\begin{array}{c} \hat{f}\left(r,\theta \right)=\frac{1}{2\pi }. \end{array}$$

Among them, ^*∗*^ is means convolution, where 1/*πx*_*r*_ is the convolution factor of Hilbert transform. The operation *∂p* of the differential operator will amplify the high-frequency noise of the signal. The Hilbert transform also has the characteristic of singularity, which causes trouble for the inverse Radon transform to directly reconstruct the CT image. Therefore, its application in practice has not yet been popularized.

In the CT imaging detection system, the distance between the detected object and the image intensifier of the imaging device is non-zero, because the size of the workpiece is used to fix the detected object, and the imaging detector in the image intensifier is inside rather than on the surface [20]. The imaging is affected by the X-ray image intensifier. The noise in the image is complex, and the image signal-to-noise ratio is low; this imaging scheme does not require a complex and sophisticated mechanical scanning structure, as shown in Figure 3.

Therefore, the electrons emitted by the X-ray cathode are not concentrated on a point on the microchannel plate but are scattered and distributed. The deviation distance of the electrons in the radial direction Δ*r* is

(12) $$\begin{array}{c} \Delta r=2d\sin\theta \sqrt{\frac{V_{0}}{V_{s}}.} \end{array}$$

The trajectory of the multiplier electrons emitted by the microchannel plate under the action of the electric field between the microchannel plate and the phosphor screen can be described by the following equation:

(13) $$\begin{array}{c} Z\left(t\right)=v_{0}*t*\cos\theta +\frac{e}{2m}*E*t^{2}. \end{array}$$

The initial kinetic energy of the multiplier electrons emitted from the microchannel plate and the velocity of the emitted electrons *v*_0_ have the following relationship:

(14) $$\begin{array}{c} eU_{0}=\frac{1}{2}mv_{0}^{2}. \end{array}$$

The scattering radius *r* of the emitted electrons to the phosphor screen relative to the axial direction is

(15) $$\begin{array}{c} r=2L\sin\theta \sqrt{\frac{U_{0}}{U}.} \end{array}$$

According to the sampling law, when the camera is used to digitally sample the visible light image on the X-ray image intensifier output phosphor screen, the following formula must be satisfied:

(16) $$\begin{array}{c} \varpi_{CMOS}\geq 2\varpi_{image}. \end{array}$$

The spatial frequency image of the image plane on the camera *ϖ* is

(17) $$\begin{array}{c} \varpi =\frac{\varpi }{M}=5lp/nm\frac{5lp}{nm}/0.1=\frac{50lp}{nm}. \end{array}$$

Then, the resolution that meets the requirements of the law is

(18) $$\begin{array}{c} \varpi_{CMOS}\geq 2\varpi =\frac{100lp}{nm}. \end{array}$$

In the X-ray imaging detection system, the total intensity of X-rays emitted by the X-ray tube is

(19) $$\begin{array}{c} I_{0}={\int^{}}_{\lambda \text{min}}^{\infty }I\left(\lambda \right)d\lambda \approx kZiV^{2}. \end{array}$$

In the formula, *λ* represents the wavelength of X-rays, *k* represents a constant, and *Z* represents the atomic number of the anode target material of the X-ray tube. It represents the current of 32 tubes of the X-ray tube, and V represents the voltage applied by the anode of the X-ray tube. The contrast of X-ray imaging detection system is

(20) $$\begin{array}{c} \Delta D=\frac{0.434\mu G\Delta T}{1+n}. \end{array}$$

In the above formula, *n* is the scattering ratio of the interaction between X-rays and the substance, where *μ* represents the ray absorption coefficient of the detected object, and Δ*T* represents the thickness of the defect. The CT value of a substance is equal to the difference between the attenuation coefficient of the substance and the absorption coefficient of water and then multiplied by the index factor after comparing with the attenuation coefficient of water. The CT value of a substance reflects the density of the substance; that is, the higher the CT value of the substance, the higher the density of the substance.

### 2.3. BPR Theory

The BPR theory is one of the most important management theories in the 1990s. It defines the banking business restructuring theory as a comprehensive business plan to assist the business in making significant progress in terms of quality, cost, service, and speed [21]. The most important thing about business process reengineering is to have a sound business process reengineering management plan and implementation steps at the executive level of the organization, as well as a clear understanding of the expected obstacles and resistance.

The main conditions for the successful implementation of BPR are as follows:

1. Change management thinking. Business process reengineering first requires all employees of the enterprise to realize a conceptual change from top to bottom [22]. Under the new business process operation mode, companies must break the previous institutions, personnel, and organizational models under the planned economy. Therefore, in the context of business process reengineering, it is necessary to actively change management thinking first.
2. Build a benign corporate culture. Business process reengineering also requires a benign corporate culture, or corporate humanistic environment. Corporate culture is the characteristic of the enterprise: the values and behaviors of the corporate group have the functions of restraint, guidance, encouragement, and cohesion. Corporate team culture will profoundly affect corporate business processes. A benign and advanced culture must promote the redesign of business processes.
3. Use advanced information technology information. Technology has a decisive effect on business process reengineering. The thinking framework of process reengineering determines the IT model. Advanced information technology is the basis for BPR to fully exert corporate efficiency.
4. Management support. Enterprise business process reengineering is a comprehensive and fundamental change. If the senior management cannot provide guarantee and support in terms of authority, business process reengineering and development will undoubtedly face difficulties [23]. The strong support of business leaders is the guarantee for business process reengineering to obtain financial and human resources support. Business managers should act as change drivers, and their beliefs and enthusiasm are the driving force for business process reengineering.

The process actually emphasizes that the work is completed in the organization's activities. Some people define a process as follows: “a process is a series of standardized activities that produce specific outputs to specific customers or markets.” A series of independent tasks constitute the simplest process, including one input and one output [24, 25]. The output is obtained after the input is transformed through the process. Generally, there are three ways of output. As an important part of a standardized and independent management theory and scientific system, business process is also an important part of ERSRC's innovative manufacturing activities. Nursing BPR is to break the barriers of the original nursing process and adopt a more realistic nursing process. The method enhances the efficiency of care specifically as shown in Figure 4.

In the empirical research of BPR theory, according to different cases, different scholars freely choose different entry points to conduct analysis and research, respectively, and put forward the skills and methods to guide enterprises to better use BPR management ideas. Such research results are mainly focusing on three aspects: the role of advanced information technology in BPR; the role of human factors (managers and employees) in the enterprise in BPR; and the role of various technical means in BPR. Among them, the role of advanced information technology in BPR is particularly important.

## 3. Experiments and Results of Thrombolytic Efficacy and Prognosis

### 3.1. Patient Information

We collected ischemic stroke patients who received intravenous thrombolysis in the green channel of stroke. Among them, there were 54 patients with thrombosis and 39 patients without thrombosis, a difference of 15; and there were 70 males and 30 females, a difference of 40. The diagnosis was clear and met the criteria for inclusion. There were no statistical differences in age and diabetes factors between the groups of patients with cerebral infarction. There were statistical differences in the comparison of general information such as gender, age, hypertension, diabetes, coronary heart disease, smoking history, and drinking history. The details are shown in Table 1.

As cerebral infarction can easily lead to depression, we compared the incidence of depression after stroke at the end of 3 months between the thrombolytic group and the nonthrombolytic group. The results showed that the proportion of patients with cerebral infarction without depression in the thrombolytic group was significantly higher than that of nonthrombolytic group. In the thrombolytic group and the nonthrombolytic group, the proportion of patients with cerebral infarction was significantly higher than that in the thrombolytic group. The specific data is shown in Table 2. In Table 2, *a* represents the number of people, and *b* represents the proportion in all patients. *c* represents the proportion in the reorganization.

Among them, in the thrombolysis group, the number of patients with mild, moderate, and severe poststroke depression at the end of 3 months was 10, 5, and 2, respectively. The incidence accounted for 8.74%, 3.88%, and 0.97% of cerebral infarction patients, accounting for thrombolysis. 16.07%, 7.14%, and 1.79% of the patients in the thrombolytic group accounted for 64.29%, 28.57%, and 7.14% of the depression patients in the thrombolytic group.

In the nonthrombolytic group, the number of patients with mild, moderate, and severe poststroke depression at 3 months was 13, 7, and 4, respectively, and the incidence accounted for 11.65%, 5.83%, and 2.91% of 103 cerebral infarction patients, respectively. 25.53%, 12.76%, and 6.38% of patients in the nonthrombolytic group accounted for 57.14%, 28.57%, and 14.28% of the depressed patients in the nonthrombolytic group. The details are shown in Figure 5.

After thrombolysis, we made statistics on whether the brain is still occluded. It can be seen from the effect of CT that the number of patients passing through the occlusion is 40, and the diagnosis of the blood flow classification of the patients after thrombolytic therapy is consistently good, as shown in Table 3.

We divided these patients into a significant improvement group and a nonsignificant improvement group. There was no statistically significant difference in age, diastolic blood pressure, systolic blood pressure, blood sugar, NIHSS baseline score, and time window between the two groups (*P* > 0.05). There was also no significant difference in gender, hyperlipidemia, hypertension, diabetes, past medical history, and smoking history (*P* > 0.05). The two groups of patients had severe ICA stenosis or occlusion, blood flow classification, vascular occlusion position, and soft. There was no significant difference in the blood supply of meningeal collateral branches (*P* > 0.05). The differences in the establishment of collateral circulation, atrial fibrillation, ulcerative plaque, and RLS between the two groups were statistically significant (*P* < 0.05) as shown in Figure 6.

### 3.2. Comparison of Treatment Effects of Patients

We first used different methods to treat different groups of patients and compared their physical recovery after treatment. We counted the changes in patients within 7 days, as shown in Figure 7.

It can be seen from Figure 7 that the patient's physical condition is not much different between the thrombolytic group and the nonthrombolytic group immediately after treatment, and the difference between the two is within 10%, but in the statistics for 7 days after treatment, the recovery of the thrombolytic group was much higher than that of the nonthrombolytic group; especially within 3 days after treatment, the brain function recovery of the thrombolytic group was more than 60% higher than that of the nonthrombolytic group, and after treatment, after 7 days, the two groups of patients stabilized, but the recovery of thrombolytic patients was still higher than that of the nonthrombolytic group.

We took care of the two groups of patients using BPR and traditional nursing methods, respectively, and then compared their physical changes and their satisfaction with nursing. Among them, the patient's physical changes are shown in Figure 8.

It can be seen from Figure 8 that, in different nursing methods, the various indicators of the patient have different changes. In the traditional nursing model, the patient takes care after the treatment, and the various indicators of the body are slightly improved, but there is still a long way to go in recovery. However, in the BPR nursing model, the patient's physical rehabilitation efficiency is greatly improved. Compared with the traditional model, the patient's bleeding is greatly reduced, and the time required for nursing is also reduced by more than 50% compared with the traditional model. We also conducted statistics on the satisfaction of different modes after nursing, and the results are shown in Figure 9.

As can be seen in Figure 9, there is a big difference in patient satisfaction among different groups. In traditional nursing, the main number of patients is distributed in general experience, while dissatisfaction accounts for about 12% of the total proportion, and satisfaction is above 32%. In the BPR nursing process, the dissatisfaction of patients is only 5%, and the proportion of patients who are satisfied or above is more than 70%. Compared with the traditional nursing model, the satisfaction is nearly 40% higher.

We count the imaging conditions of patients with different degrees of cerebral infarction under CT images, and CT imaging can more clearly understand the performance characteristics of different degrees of cerebral infarction, as shown in Figure 10.

In univariate analysis related to thrombolytic efficacy, hyperlipidemia, atrial fibrillation, M1 occlusion, establishment of collateral circulation, ulcerative plaque, and right-to-left shunt were *P* < 0.1, which were included in the multivariate analysis. The logistic regression analysis showed that right-to-left shunt and establishment of collateral circulation were independent predictors of significant improvement after intravenous thrombolysis (*P* < 0.05). The results are shown in Table 4.

## 4. Discussion

### 4.1. Cerebral Infarction

The stenosis or occlusion of large atherosclerosis can lead to large-scale cerebral infarction. A large number of brain cells are due to ischemia and hypoxia, tissue metabolism disorder, neurological dysfunction, clinically mainly manifested as hemiplegia, hemisensory disorder, hemianopia, impaired consciousness, language disorder, and other symptoms, if cerebral edema occurs in the infarcted hemisphere, it will also cause midline shift and brain herniation. In severe cases, it can be life-threatening and is the most serious type of ischemic stroke. In this study, CT images were selected to observe the nursing BPR to observe the thrombolytic efficacy and prognosis of patients with cerebral infarction. From the results, it can be seen that it is particularly important to restore blood perfusion as soon as possible within the time window. Thrombolytic therapy with recombinant tissue plasminogen activator in the acute phase, hyperacute phase, and acute phase is safe, simple, and effective. It has become the first-line treatment method for acute ischemic stroke. CT imaging and reasonable nursing can help the local blood supply in the “ischemic penumbra” area quickly restored, which significantly improves tissue metabolism, improves brain tissue function, saves surviving neurons to the greatest extent, and fully restores the physiological functions of nerve cells.

From the experimental results, it can be shown that intravenous thrombolysis using rt-PA within 4.5 hours of onset or in line with imaging thrombolysis standards can recanalize blood vessels and recover the symptoms of neurological deficits in most patients. The comparison of blood flow score and patient scores shows that the improvement of MCA blood flow score shown by TCD is basically the same as the improvement of NIHSS score. It is inferred that the blood vessels of the occluded patients are reperfused after reperfusion therapy, and the brain is in the ischemic penumbra. Neuronal activity recovered after tissue reperfusion, so the patient's clinical symptoms disappeared or improved, and the score decreased. Therefore, for ischemic stroke, the principle of early detection and early treatment should be followed.

### 4.2. Clinical Nursing

It can be seen that CT imaging has high specificity and good reliability in diagnosing stenosis and occlusion of the main intracranial artery. It can accurately assess the degree of recanalization of the responsible artery and help determine the prognosis of patients receiving thrombolytic therapy. For patients with cerebral infarction, from the experimental record, traditional nursing methods are not satisfactory. Traditional nursing costs a lot and consumes a lot of time, but the nursing effect is unsatisfactory. This article compares BPR nursing with traditional nursing, by observing and analyzing the blood flow velocity, spectrum shape, vascular pulsation index in multiple depths, and obtaining a more complete blood flow by analyzing the hemodynamic changes in the proximal and distal segments of the occluded blood vessel. Information about the use of BPR care can not only comprehensively evaluate the blood flow velocity, spectrum shape, and *P* value of the responsible artery, but also provide quantitative standards for research and improvement of the operability of experimental data. Therefore, BPR observation nursing has a high accuracy rate in the diagnosis of vascular stenosis and occlusion and is convenient for bedside operation and dynamic observation. It can be widely used in the diagnosis and treatment of intravenous thrombolysis in patients with ischemic stroke. This paper found that the difference between the significantly improved group and the unremarkably improved group in severe stenosis or occlusion of the internal carotid artery was not statistically significant, while the difference in ulcerative atherosclerotic plaque was statistically significant.

With the aid of assessing the establishment of collateral circulation and the diagnosis of carotid ulcerative atherosclerotic plaque, the above imaging characteristics are related to the efficacy of intravenous thrombolytic therapy in patients with IS; in the multivariate logistic regression analysis, the BPR observation, the establishment of collateral circulation in nursing assessment, and RLS diagnosed by c-TCD are independent predictors related to significant improvement after intravenous thrombolysis. These two imaging examinations have certain value in predicting the effect of intravenous thrombolysis.

## 5. Conclusion

In this article, CT imaging examination is used as a means to diagnose patients with cerebral infarction. At this time, the patient's intravenous thrombolytic therapy has been started. This can quickly check the target blood vessel at the bedside of the neuro-intensive care unit. On the one hand, it is for patients with a clear time window. Start intravenous thrombolytic therapy as soon as possible to minimize unnecessary hospital delays and save the brain tissue to the greatest extent. Inspection of occluded arteries through BPR care can also improve the efficiency of intravenous thrombolysis and improve the prognosis of patients with ischemic stroke. Of course, this article also has some shortcomings due to objective factors such as conditions and time, because patients with ischemic stroke often have disturbances in consciousness, speech, or other discomforts and often cannot cooperate, especially after intravenous thrombolysis. Patients in the group may be more likely to be unable to cooperate with movements due to poor recovery of neurological function. In addition, the design of this study included only the clinical and imaging data of the enrolled subjects after 7 days of intravenous thrombolytic therapy. The long-term prognostic data such as the review data after 3 months and the follow-up visit information were not included in the scope of the study, making the experiment and results have certain limitations. In future research, the details and feasibility of the entire operation process should be considered more comprehensively and carefully to avoid improper situations where patients cannot cooperate and have no alternative means.

## Figures and Tables

**Figure 1:** CT radiography system structure.

**Figure 2:** Schematic diagram of ray attenuation passing through an object.

**Figure 3:** Schematic diagram of the imaging detection system.

**Figure 4:** Nursing flow chart.

**Figure 5:** Depression levels in different groups.

**Figure 6:** Statistical differences between different groups of patients.

**Figure 7:** Treatment effect of different groups of patients.

**Figure 8:** Effects of different care methods.

**Figure 9:** Satisfaction survey results.

**Figure 10:** Different situations of patients with cerebral infarction.

**Table 1:** Patient data statistics.

Project	Thrombolysis group	Nonthrombolytic group	*χ* ^2^/*t*	*P*
Gender (male female)	38/16	32/17	0.148	0.583
Age	62.28 ± 8.33	65.37 ± 12.17	0.468	0.625
Hypertension (yes/no)	31/24	33/14	0.817	0.356
Diabetes (yes/no)	11/47	12/38	1.425	0.243
Coronary heart disease (yes/No)	16/41	14/35	0.283	0.579
Smoking (yes/no)	23/34	12/35	2.423	0.127
Drinking (yes/no)	16/59	11/47	2.173	0.132

**Table 2:** Proportion of suppression caused by cerebral infarction.

Group	Thrombolysis group			Nonthrombolytic group			Total	Incidence
	*a*	*b*	*c*	*a*	*b*	*c*		
No depression	43	41.56%	74.69%	25	24.27	54.31%	68	64.76%
Depression	15	14.12%	24.68%	22	21.57	43.57%	37	35.24%
Total	58	—	—	47	—	—	105	100%

**Table 3:** Scores of patients with occlusion after thrombolysis.

	Vascular occlusion	Partial recanalization of blood vessels	Complete recanalization of blood vessels	Total
Vascular occlusion	24	3	1	28
Partial recanalization of blood vessels	0	15	4	19
Complete recanalization of blood vessels	0	3	52	55
Total	24	21	57	102

**Table 4:** Multivariate analysis related to the efficacy of intravenous thrombolysis.

	95% CI	OR	*P*
Hyperlipidemia	0.405–3.463	1.247	0.424
Collateral circulation established	1.157–82.733	9.496	0.033
Atrial fibrillation	0.124–1.098	0.354	0.089
M1 occlusion	0.594–4.721	1.608	0.298
Ulcerative plaque	0.824–7.054	2.361	0.097
Right to left diversion	2.131–16.258	5.932	0.001

## Data Availability

The data that support the findings of this study can be obtained from the corresponding author upon reasonable request.
